The article "Up-regulation of miRNA-148a inhibits proliferation, invasion, and migration while promoting apoptosis of cervical cancer cells by down-regulating RRS1" was retracted in 2020. Reasons: manipulated images; duplicated images.

# Up-regulation of miRNA-148a inhibits proliferation, invasion, and migration while promoting apoptosis of cervical cancer cells by down-regulating RRS1

**DOI:** 10.1042/BSR20181815

**Published:** 2019-05-07

**Authors:** Ying Zhang, Bingmei Sun, Lianbin Zhao, Zhengling Liu, Zonglan Xu, Yonghui Tian, Changhong Hao

**Affiliations:** 1 Department of Obstetrics and Gynecology, Linyi Central Hospital, Linyi 276400, Shandong Province, P.R. China; 2 Department of Emergency, Linyi Central Hospital, Linyi 276400, Shandong Province, P.R. China

**Keywords:** Cervical cancer, Invasion, microRNA-148a, Migration, Proliferation, RRS1

## Abstract

The purpose of the present study is to figure out the role of miRNA-148a (miR-148a) in growth, apoptosis, invasion, and migration of cervical cancer cells by binding to regulator of ribosome synthesis 1 (RRS1). Cervical cancer and adjacent normal tissues, as well as cervical cancer cell line Caski, HeLa, C-33A, and normal cervical epithelial cell line H8 were obtained to detect the expression of miR-148a and RRS1. Relationship between miR-148a and RRS1 expression with clinicopathological characteristics was assessed. The selected Caski and HeLa cells were then transfected with miR-148a mimics, miR-148a inhibitors or RRS1 siRNA to investigate the role of miR-148a and RRS1 on proliferation, apoptosis, colony formation, invasion, and migration abilities of cervical cancer cells. Bioinformatics information and dual luciferase reporter gene assay was for used to detect the targetting relationship between miR-148a and RRS1. Down-regulated miR-148a and up-regulated RRS1 were found in cervical cancer tissues and cells. Down-regulated miR-148a and up-regulated RRS1 are closely related with prognostic factors of cervical cancer. RRS1 was determined as a target gene of miR-148a and miR-148a inhibited RRS1 expression in cervical cancer cells. Up-regulation of miR-148a inhibited cell proliferation, migration, and invasion while promoting apoptosis in Caski and HeLa cells. Our study suggests that miR-148a down-regulates RRS1 expression, thereby inhibiting the proliferation, migration, and invasion while promoting cell apoptosis of cervical cancer cells.

## Introduction

Cervical cancer is known as the third most common cancer and the fourth leading reason of cancer-related death in female in the world [1]. Statistics show that more than 50,000 females succumb to cervical cancer each year in China [2]. Although it is reported that 99.7% of patients with cervical cancer could be resulted from long-term infection in high-risk human papillomaviruses [3], other factors, such as host and viral genetic factors, are also implicated in the development of cervical cancer [4]. In recent decades, great advances have been achieved in surgery, irradiation, as well as chemotherapy for the treatment of cervical cancer, but the prognosis of patients with cervical cancer remains to be unsatisfactory owing to late diagnosis [5, 6]. Except that, the specific molecular mechanisms referring to the initiation and progression of cervical cancer are still unknown. Based on this, better understanding the mechanisms for the occurrence and progression of cervical cancer will help to seek for the novel biomarkers and treatment targets, all of which is pivotal for improving the prognosis of patients with cervical cancer.

Recently, [7] emerging evidence has also revealed that alterations in (miRNAs) are participated in the development, progression as well as metastasis in tumors [8]. As previously reported, abnormally expressed miRNAs are found in many types of human cancers, which function as either tumor promoters or suppressors based upon the nature of their targets [9]. MiR-148 was proved to play an important role in regulating immune balance and antigen presentation and inhibiting the production of numerous inflammation-associated cytokines [10–12]. Meanwhile, recent evidence has suggested that miR-148a was aberrantly expressed in different types of cancers, which might act as an either oncogene or tumor suppressor and also play essential roles in the potential mechanisms in oncogenesis [13–16]. A previous study has indicated that HOTAIR may act as an endogenous sponge to control the expression of HLG-A via competitively targetting miR-148a in cervical cancer cells [17]. Regulator of ribosome synthesis 1 (RRS1) was initially discovered in yeast that consisting of 203 amino acids [18], which is also a conserved nuclear protein in eukaryotes [19]. Additionally, RRS1 is an important protein acting as a linker between ribosome biogenesis and protein secretion [20, 21]. Gambe et al. silenced the RRS1 gene in cervical cancer heLa cells by RNA interference technique and then found that the number of cells in tetraploid stage increased and the cell division time was prolonged [22], suggesting its regulatory role in disease and tumorigenesis and development. However, no study focussed on the role of miR-148a and RRS1 in the initiation and progression of cervical cancer. In view of this, we performed the present study to figure out the role of miR-148a in growth, apoptosis, invasion, and migration of cervical cancer cells by binding to RRS1.

## Materials and methods

### Ethics statement

The study adhered to the tenets of the World Medical Association Declaration of Helsinki, and it was approved by the regional Ethics Committee of Linyi Central Hospital. Patients should have a full understanding of the study, the ability to complete all treatment plans, and sign the relevant informed consent.

### Study subjects

From September 2016 to December 2017, the cervical cancer tissues and the corresponding adjacent normal tissues were collected from 114 patients with cervical cancer (aged from 32 to 68 years, with an average age of [45.5 ± 7.2] years) in Linyi Central Hospital. All patients were not treated with radiotherapy and chemotherapy, and had complete clinical data. The inclusion criteria were: all patients should have histopathological results; the diagnostic criteria of cervical cancer based on the sixth edition of the Diagnostic Criteria of Gynecology and Obstetrics; staging for patients were based on FIGO staging criteria of the International Federation of Obstetrics and Gynecology [23]; women who need or require radical hysterectomy; and patients were postoperatively confirmed by pathology. The exclusion criteria were: patients with incomplete clinical data; and patients with congenital acute genital tract inflammation, pregnancy, hereditary diseases, and severe internal diseases. The selected adjacent normal tissues were tissues that near the cervical cancer tissues with no cancer tissue found under the microscope. All diagnoses were made by pathologists. Cervical cancer tissues or adjacent normal tissues (about 0.5 mm^3^) were collected immediately after operation. After that, those tissues were immediately rinsed with normal saline to remove blood, placed in a tissue cryopreservation tube, immediately put in liquid nitrogen for 1 h, and then moved to −80°C refrigerator for preservation until use.

### Cell culture

Cervical cancer cell line Caski, HeLa and C-33A as well as normal cervical epithelial cell line H8 purchased from the Cell Resource Center of Shanghai Institutes for Biological Sciences (Chinese Academy of Sciences, Shanghai, China) were cultured in RPMI1640 medium containing 10% fetal bovine serum (FBS), 100 U/ml penicillin and 100 μg/ml streptomycin in an incubator with a volume fraction of 5% CO_2_ at 37°C. When the cell confluency was over 80%, the cells were detached with 0.25% trypsin and subcultured according to the need of the experiment. The cells in logarithmic growth period were selected for the following experiments.

### Cell grouping and transfection

Caski and HeLa cells were classified into blank group (without transfected with any sequence), mimics negative control (NC) group (cells transfected with mimics NC plasmid), miR-148a mimics group (cells transfected with miR-148a mimics plasmid), inhibitors NC (cells transfected with inhibitors NC plasmid), miR-148a inhibitors group (cells transfected with miR-148a inhibitors plasmid), miR-148a inhibitors + siRNA-NC (cells transfected with miR-148a inhibitors and siRNA-NC plasmid), miR-148a inhibitors + RRS1 siRNA (cells transfected with miR-148a inhibitors and siRNA-RRS1 plasmid) and RRS1 siRNA group (cells transfected with siRNA-RRS1 plasmid). The above oligonucleotide sequences are purchased from Shanghai GenePharma Co., Ltd (Shanghai, China). The Caski and HeLa cells in logarithmic growth phase were obtained and transfected with the sequences of mimics NC, miR-148a mimics, inhibitors NC, miR-148a inhibitor, miR-148a inhibitors + siRNA-NC, miR-148a inhibitors + RRS1 siRNA and RRS1 siRNA according to the instructions of Lipofectamine™ 2000 (Invitrogen Corp., Carlsbad, CA, U.S.A.). The cell concentration of each group was adjusted to 5 × 10^4^ per ml, and the cells were inoculated in a six-well cell culture plate (2 ml in each well) for culturing in a 5% CO_2_ incubator at 37°C. When the cell confluency reached 30–50%, cell transfection was performed. After transfection, the cells were placed at room temperature for 20 min. After 6 h, the original culture medium was replaced with RPMI1640 culture medium for another 48 h culturing.

### Dual-luciferase reporter gene assay

The binding site of RRS1 and miR-148a was determined by online prediction software http://www.targetscan.org. The synthetic primers were designed based on the 3′-UTR sequence of RRS1 gene, and the restriction endonuclease Hind III and Spe I sites were introduced into the forward and reverse primers, respectively, and the mutation sequence of the binding site was designed. The target sequence fragment was synthesized by GenScript Biotech Corp., Nanjing, China). The target product and pMIR-REPORT™ Luciferase vector plasmids were digested by restriction endonuclease Hind III and Spe I. The digested products were recycled and ligated with T4 DNA ligase to transform DH5α competent Escherichia coli. The recombinant plasmid was identified by enzyme digestion and sequencing. In the 12-well plate, 1 × 10^5^ Caski and HeLa cells were seeded into each well. The cells were co-transfected with the recombinant plasmid and miR-148a mimics for 48 h according to the corresponding groups and then washed with PBS three times after abandoning the cell culture medium. Cell lysis solution (100 μl) of luciferase kit was added in each well for lysis for 30 min. Cell lysis solution (20 μl) was added with 100 μl LAR II, which was used to measure fluorescence value (A), and cell lysis solution was added with 100 μl Stop&Glo reagent to measure fluorescence value (B). Fluorescence value (A) of firefly was used as an internal reference to calculate luciferase activity.

### Reverse transcription quantitative PCR

TRIzol method (Takara Biomedical Technology [Dalian] Co., Ltd) was adopted for extracting the total RNA in cells and tissues in order to determine the concentration and purity of RNA. The sample RNA was reversed to cDNA based on the instructions of the Reverse Transcription Kit (DRR047S, Takara Biomedical Technology [Dalian] Co., Ltd), with the total system being 10 μl. The obtained cDNA was added with 65 μl diethyl pyrocarbonate (DEPC) water to dilute and mix well. The RT-PCR reaction system was prepared based upon the following components: 5 μl of SsoFast EvaGreen Supermix (1708882, Bio-Rad, CA, U.S.A.), 0.5 μl of Forward primer (10 μM), 0.5 μl of Reverse primer (10 μM), and 4 μl cDNA. The PCR amplification conditions were predenatured at 95°C for 1 min, followed by 30 cycles of denaturing at 95°C for 30 s, annealing at 58°C for 5 s, and finally extending for 5 s. The primers were synthesized by Shenzhen Huada Gene Co., Ltd. (Shenzhen, Guangdong, China). U6 or glyceraldehyde-3-phosphate dehydrogenase (GAPDH) was used as an internal reference, with six parallel wells set for per gene in each sample. The reliability of PCR results was evaluated by the dissolution curve, and the CT value (inflection point of the expanded dynamic curve) was taken. △Ct = CT_(target gene)_ − CT_(internal reference)_, △△Ct = △Ct_(experimental group)_ − △Ct_(control group)_. The relative expression of target gene was calculated by 2^−△△*C*^_T_ [24]. The experiment was repeated three times.

### Western blot analysis

The total protein was extracted from the tissues and cells of each group. Bicinchoninic acid (BCA) protein concentration assay kit was used to measure protein concentration, and the protein concentration of each group was adjusted. After adding with 5× SDS loading buffer, the cells were denatured at 95°C for 5 min, separated by SDS-PAGE, and transferred into membrane. After that, the membrane was added with 5% skim milk powder for sealing overnight at 4°C. After the membrane was washed with Tris-buffered saline, 1% Tween 20 (TBST), it was then added with the primary antibody RRS1 (1:1000, Abcam, U.K.), and GAPDH (1:1000, Millipore Inc., U.S.A.) for incubation overnight at 4°C. After the membrane was washed with TBST again, it was then added with horse radish peroxidase (HPR)-labeled secondary antibody (Abcam, U.K.) for incubation overnight at 4°C. After the membrane was washed with TBST, enhanced chemiluminescence was used for developing. The gray value of the target band was analyzed by ImageJ software, and the experiment was repeated three times independently.

### MTT assay

When the transfected Caski and HeLa cells reached 80% confluency, the cells were washed with PBS twice, detached by routine trypsin, and triturated into the single cell suspension by the straw. The counted cells were inoculated in a 96-well plate, 3 × 10^3^ – 6 × 10^3^ cells were inoculated in each well, with 200 μl in each well, for incubation in a 5% CO_2_ incubator at 37°C for 24–72 h. Six parallel wells were set. After that, 20 μl of MTT solution (5 mg/ml, Sigma–Aldrich, St. Louis, MO, U.S.A.) was added to each well for coloration. Next, the culture was terminated and the culture medium was abandoned after incubating in a 5% CO_2_ incubator at 37°C for 4 h. Each well was added with DMSO (150 μl), shaking gently for 10 min to induce crystallization dissolution. The optical density (OD) value of each well was determined by a microplate reader at 0, 24, 48, and 72 h, respectively. With OD value set as ordinate, and the interval time as horizontal ordinate, a MTT curve was constructed. The experiment was independently repeated three times.

### Colony formation assay

After 72 h of transfection, the cells in logarithmic growth phase were inoculated in a six-well culture plate, with 200 cells per well. Six parallel wells were set up and in stationary culture for 2 weeks. When white clone spots can be seen with the naked eye, the culture was terminated. After that, the cells were fixed with methanol (2 ml) at room temperature for 15 min, then stained with Giemsa solution at room temperature for 15 min, washed with running water slowly and dried. Cell clones with more than 50 cells were counted under an optical microscope for calculating the colony formation rate, which was calculated as the number of cloned cells/inoculated cells × 100%. The experiment was repeated three times.

### Flow cytometry

The cells were seeded into a six-well culture plate according to 1 × 10^6^ cells per well. Cells were cultured synchronously for 12 h after cell adhesion, the original culture medium was discarded and the corresponding treatment was given for a specific time. Cells were collected by centrifugation after detachment of cells, which were washed with PBS twice, resuspended with precooled 75% ethanol and fixed overnight at −20°C. After centrifugation, the supernatant was abandoned. The cells were rinsed with PBS twice. In each sample, 450 μl of PBS was used to suspend cells. After that, the cells were added with 50 μl of propidium iodide (PI, 0.5 mg/ml), then mixed together, and placed in 37°C water-bath for 30 min. After centrifugation, the supernatant was discarded and the cells were suspended with PBS. Cell cycle distribution was measured and analyzed by flow cytometer BD FACSAria™ cell sorter (BD Biosciences, San Jose, CA, U.S.A.). The experiment was repeated three times independently.

After 72 h of transfection, the collected cells were rinsed with PBS three times and then added to the precooled 1 × binding buffer (500 μl). Next, the cell suspensions were added with 5 μl of Annexin-V-FITC and 2.5 μl of PI and mixed gently. The cell apoptosis was determined by flow cytometer BD FACSAria™ cell sorter (BD Biosciences, San Jose, CA, U.S.A.). In the scattered plot, the lower left quadrant (Q4) showed healthy living cells (FITC^−^/PI^−^), the lower right quadrant (Q3) showed early apoptotic cells (FITC^+^/PI^−^), the right upper quadrant (Q2) showed necrosis, and late apoptosis cells (FITC^+^/PI^+^). The apoptosis rate was calculated as early apoptosis percentage (Q3) + late apoptosis percentage (Q2). The experiment was repeated three times independently.

### Scratch test

The scratches with an interval of 0.5–1.0 cm were made by a marker pen at the back of the six-well plate, which perpendicular is to the horizontal axis. Cells at logarithmic growth period were treated with serum-free medium for 12–24 h and then inoculated into a six-well plate with 5 × 10^5^ cells per well. When the cell confluency reached 90%, the cells were scratched along the marking line using a gun head perpendicular to the plate and washed twice with PBS to remove the floating cells. The cells were supplemented with McCoy s5a medium and cultured in a saturated humidity with 5% CO_2_ at 37°C. Photographs were taken under an inverted microscope at 0 and 24 h. Image tool software (Bechtel Nevada, Los Alamos Operations) was used to calculate healing area, which was calculated as (width value of initial scratch − width value of current scratch)/width value of initial scratch × 100%. The experiment was repeated three times.

### Transwell assay

Preparation of single cell suspension from serum-free medium was conducted by conventional method, with 5 × 10^5^ cells per milliliter. Matrigel was dissolved overnight at 4°C, which was diluted with serum-free DMEM medium at the ratio of 1:3, and 30 μl diluted Matrigel was added into the apical chamber in each Tanswell chamber for three times (15, 7.5, and 7.5 μl) (Corning, NY, U.S.A.). At intervals of 10 min, the Matrigel was evenly spread and all micropores on the bottom of the apical chamber were covered. The DMEM medium containing 10% FBS was added to the basolateral chamber of the 24-well plate with the cell suspensions inoculated into the apical chamber of Transwell. The number of cells passing through the Matrigel was used as an indicator of invasion. The experiment was repeated three times.

### Statistical analysis

SPSS 19.0 (SPSS Inc, Chicago, IL, U.S.A.) software was used for data analyzing, and the experiment was repeated three times independently to calculate mean and S.D. The measurement data were expressed as mean and S.D. The *t* test was used to analyze the difference between groups. One-way analysis of variance was used to analyze the difference amongst three or more groups. Bilateral analysis was used in all analyses, and significant differences were observed in *P*<0.05. Table 1.

**Table 1:** Primer sequences

	Primer sequences (5′- 3′)
miR-148a	Forward: 5′-ACACTCCAGCTGGGTCAGTGCACTACAGAA-3′
	Reverse: 5′-CTCAACTGGTGTCGTGGAGTCGGCAATTCAGTTGAGACAAAGTT-3′
U6	Forward: 5′-CTCGCTTCGGCAGCACA-3′
	Reverse: 5′-AACGCTTCACGAATTTGCGT-3′
RRS1	Forward: 5′-CCCTACCGGACACCAGAGTAA -3′
	Reverse: 5′-CCGAAAAGGGGTTGAAACTTCC-3′
GAPDH	Forward: 5′-AACGGATTTGGTCGTATTGGG-3′
	Reverse: 5′-TCGCTCCTGGAAGATGGTGAT-3′

## Results

### Down-regulated miR-148a and up-regulated RRS1 are found in cervical cancer tissues

Reverse transcription quantitative PCR (RT-qPCR) was used to detect the miR-148a expression and RRS1 mRNA expression in cervical cancer and adjacent normal tissues. Meanwhile, western blot analysis was used to detect the protein expression of RRS1 in cervical cancer tissues and adjacent normal tissues. As shown in the results of RT-qPCR (Figure 1A), the miR-148a expression in cervical cancer tissues was (0.144 ± 0.018), which was significantly lower than that in adjacent normal tissues (1.000 ± 0.002) (*P*<0.05). RRS1 mRNA expression in cervical cancer tissues was (3.892 ± 0.104), which was significantly higher than that in adjacent normal tissues (1.000 ± 0.003) (*P<*0.05). As shown in the results of western blot analysis (Figure 1B,C), RRS1 protein expression in cervical cancer tissues was (0.965 ± 0.073), which was significantly higher than that in adjacent normal tissues (0.458 ± 0. 034) (*P<*0.05). Correlation analysis of the expression of miR-148a and RRS1 in cervical cancer tissues showed that there was a significant negative correlation between the two (r = –849; *P<*0.05).

**Figure 1:** Down-regulated miR-148a and up-regulated RRS1 are found in cervical cancer tissues (**A**) miR-148a expression and RRS1 mRNA expression in cervical cancer and adjacent normal tissues; (**B,C**) protein expression of RRS1 in cervical cancer and adjacent normal tissues.

### Down-regulated miR-148a and up-regulated RRS1 are closely related with prognostic factors of cervical cancer

The expression of miR-148a was ranked from high to low, and the expression of miR-148a was divided into two levels: high and low with the 75th percentile level as the critical point [25]. Amongst 114 patients, there are 30 patients had up-regulated miR-148a expression, and 84 patients had down-regulated miR-184a expression. Relationship between miR-148a expression and clinicopathological characteristics is shown in Table 2. The low expression of miR-148a was significantly correlated with FIGO stage, lymph node metastasis and vascular invasion (*P<*0.05), while no significant difference was found between low expression of miR-148a and age, differentiation degree, and tumor size (*P>*0.05). The expression of RRS1 was ranked from high to low, and the expression of RRS1 was divided into two levels: high and low with the 75th percentile level as the critical point [25]. Amongst 114 patients, there are 76 patients had up-regulated RRS1 expression, and 38 patients had down-regulated RRS1 expression. Relationship between RRS1 expression and clinicopathological characteristics is shown in Table 2. The high expression of RRS1 was significantly correlated with FIGO stage, lymph node metastasis, and vascular invasion (*P<*0.05), while no significant difference was found between low expression of RRS1 and age, differentiation degree and tumor size (*P*>0.05). The results suggested that down-regulated miR-148a and up-regulated RRS1 are closely related with prognostic factors of cervical cancer.

**Table 2:** Relationship between miR-148a and RRS1 expression with clinicopathological characteristics

Clinicopathological characteristics	cases	miR-148a expression		*P*	RRS1 mRNA expression		*P*
		Low	High		Low	High	
Age				0.656			0.536
≤45 years	40	31	9		15	25	
>40 years	74	53	21		23	51	
FIGO stage				0.016			0.007
IB1/IB2	83	56	27		34	49	
IIA	31	28	3		4	27	
Lymph node metastasis				0.023			0.003
No	95	66	29		37	58	
Yes	19	18	1		1	18	
Vascular invasion				0.031			0.015
No	68	45	23		29	39	
Yes	46	39	7		9	37	
Differentiation degree				0.099			0.145
Well	15	10	5		8	7	
Moderate	84	66	18		24	60	
Poor	15	8	7		6	9	
Tumor size				0.232			0.268
≤4cm	83	64	19		25	58	
>4cm	31	20	11		13	18	

### Down-regulated miR-148a and up-regulated RRS1 are found in cervical cancer cells

RT-qPCR was used to detect the miR-148a expression and RRS1 mRNA expression in cervical cancer cells and normal cervical epithelial cell. Meanwhile, western blot analysis was used to detect the protein expression of RRS1 in cervical cancer cells and normal cervical epithelial cell. As shown in Figure 2A, the expression of miR-148a in the cervical cancer cell line Caski, HeLa, and C-33A was lower than that in the normal epithelial cell line H8 (*P<*0.05). The miR-148a expression in H8 was set to 1, and the relative expression of miR-148a was (0.713 ± 0.052) in Caski cells, (0.284 ± 0.038) in HeLa cells and (0.439 ± 0.042) in C-33A cells. MiR-148a expression was the lowest in HeLa cells and the highest in Caski cells. As shown in Figure 2A–C, the mRNA and protein expression of RRS1 in the cervical cancer cell line Caski, HeLa, and C-33A was higher than that in normal cervical epithelial cell H8 (*P<*0.05). RRS1 expression was the highest in HeLa cells and lowest in Caski cells. Therefore, Caski and HeLa cells were selected for further experiment.

**Figure 2:** Down-regulated miR-148a and up-regulated RRS1 are found in cervical cancer cells (**A**) miR-148a expression and RRS1 mRNA expression in cervical cancer cells and normal cervical epithelial cell; (**B,C**) protein expression of RRS1 in cervical cancer cells and normal cervical epithelial cell. * *P*<0.05 versus normal cervical epithelial cell H8. The data represent the mean ± S.D. of the three independent experiments.

### RRS1 is a target gene of miR-148a

The target site of RRS1 and miR-148a was determined by online prediction software TargetScan. The sequence of the 3′-UTR region of RRS1 mRNA combined with miR-148a is shown in Figure 3A. In order to prove that the predicted binding sites of miR-148a caused the change of luciferase activity, mutation type (Mut) sequence and wild-type (Wt) sequence of RRS1 3′UTR with the deletion of miR-148a binding site were designed respectively. Using luciferase activity assay, Caski and HeLa cells were co-transfected with the recombinant plasmids of miR-148a mimics, Wt-miR-148a/RRS1 or Mut-miR-148a RRS1, respectively. The results showed that the luciferase activity of Mut-miR-148a/RRS1 plasmid was not significantly affected by miR-148a mimics in Caski and HeLa cells, but the luciferase activity in Wt-miR-148a/RRS1 plasmid was obviously decreased affected by miR-148a mimics in Caski and HeLa cells (Figure 3B).

**Figure 3:** RRS1 is a target gene of miR-148a (**A**) TargetScan prediction of target sites for RRS1 and miR-148a; (**B**) double luciferase reporter gene assay was performed in Caski and HeLa cells. The data represent the mean ± S.D. three independent experiments.

### miR-148a inhibits RRS1 expression in cervical cancer cells

RT-qPCR was applied to detect the miR-148a expression and RRS1 mRNA expression, and western blot analysis was conducted to detect the RRS1 protein expression after transfection. In Caski and HeLa cells, in contrast with the blank, mimics NC, and inhibitors NC groups, the expression of miR-148a was increased (Figure 4A,D) in the miR-148a mimics group while the mRNA (Figure 4A,D) and protein (Figure 4B–F) expression of RRS1 was decreased in the miR-148a mimics and RRSI siRNA groups (all *P<*0.05); expression of miR-148a was decreased (Figure 4A,D), while the mRNA (Figure 4A,D) and protein (Figure 4B–F) expression of RRS1 was increased in the miR-148a inhibitors and miR-148a inhibitors + siRNA-NC groups (all *P<*0.05). In comparison with the miR-148a inhibitors + siRNA-NC group, expression of miR-148a (Figure 4A,D) showed no change while the mRNA (Figure 4A,D) and protein (Figure 4B–F) expression of RRS1 was decreased in the miR-148a inhibitors + RRS1 siRNA group (*P<*0.05; Figure 4). Compared with the miR-148a inhibitors + RRS1 siRNA group, the expression of miR-148a was increased (Figure 4A,D) in the miR-148a mimics group while the mRNA (Figure 4A,D) and protein (Figure 4B–F) expression of RRS1 was decreased in the RRS1 siRNA group (all *P<* 0.05). In Caski and HeLa cells, up-regulation of miR-148a inhibited RRS1 expression, and down-regulated miR-148a increased RRS1 expression.

**Figure 4:** In Caski and HeLa cells, up-regulation of miR-148a inhibited RRS1 expression (**A**) miR-148a expression and RRS1 mRNA expression in Caski cells; (**B**) Protein bands of RRS1 in Caski cells; (**C**) protein expression of RRS1 in Caski cells; (**D**) miR-148a expression and RRS1 mRNA expression in HeLa cells; (**E**) protein bands of RRS1 in HeLa cells; (**F**) protein expression of RRS1 in HeLa cells; *P<0.05 versus the blank, mimics NC, or inhibitors NC groups; #*P*<0.05 versus the miR-148a inhibitors + siRNA-NC group; &*P*<0.05 versus the miR-148a inhibitors + RRS1 siRNA group; there are six parallel wells in each experiment; the data represents the mean ± S.D. of the three independent experiments.

### Up-regulation of miR-148a inhibits proliferation of Caski and HeLa cells

At 0, 24, 48, and 72 h after Caski and HeLa cells were transfected, cell proliferation was detected by MTT assay (Figure 5). After Caski and HeLa cells were transfected with 48 and 72 h, in contrast with the blank, mimics NC, and inhibitors NC groups, decreased proliferation of Caski (Figure 5A) and HeLa (Figure 5B) cells was found in the miR-148a mimics and RRS1 siRNA group while increased cell proliferation was found in the miR-148a inhibitors and miR-148a inhibitors + siRNA-NC groups (all *P<*0.05). No significant difference was found in cell proliferation amongst the blank, mimics NC, and inhibitors NC groups (*P*>0.05). In comparison with miR-148a inhibitors + siRNA-NC group, decreased cell proliferation was found in the miR-148a inhibitors + RRS1 siRNA group (*P<*0.05). Compared with the miR-148a inhibitors + RRS1 siRNA group, the RRS1 siRNA group showed decreased cell proliferation (*P<*0.05). It is suggested that up-regulation of miR-148a inhibits proliferation of Caski and HeLa cells.

**Figure 5:** Up-regulation of miR-148a inhibits proliferation of Caski and HeLa cells (**A**) Comparison of Caski cell proliferation results in each group; (**B**) Comparison of HeLa cell proliferation results in each group; *P<0.05 versus the blank, mimics NC, or inhibitors NC groups; #*P<*0.05 versus the miR-148a inhibitors + siRNA-NC group; &*P<*0.05 versus the miR-148a inhibitors + RRS1 siRNA group; there are six parallel wells in each experiment; the data represent the mean ± S.D. of the three independent experiments.

### Up-regulation of miR-148a inhibits colony formation ability of Caski and HeLa cells

Colony formation ability of Caski (Figure 6A) and HeLa (Figure 6B) cells was assessed by colony formation assay. In Caski (Figure 6C) and HeLa (Figure 6D) cells, in contrast with the blank, mimics NC, and inhibitors NC groups, decreased colony formation ability of Caski and HeLa cells was found in the miR-148a mimics and RRS1 siRNA groups while increased colony formation ability was found in the miR-148a inhibitors and miR-148a inhibitors + siRNA-NC groups (all *P<*0.05). No significant difference was found in colony formation ability amongst the blank, mimics NC, and inhibitors NC groups (*P*>0.05). In comparison with the miR-148a inhibitors + siRNA-NC group, decreased colony formation ability was found in the miR-148a inhibitors + RRS1 siRNA group (*P*<0.05). Compared with the miR-148a inhibitors + RRS1 siRNA group, the RRS1 siRNA group showed decreased colony formation ability (*P*<0.05). These results suggested that in up-regulation of miR-148a could inhibit colony forming ability of Caski and HeLa cells.

**Figure 6:** Up-regulation of miR-148a inhibits colony formation ability of Caski and HeLa cells (**A**,**B**). Comparison of colony formation ability of Caski cells in each group; (**C**,**D**) comparison of colony formation ability of HeLa cells in each group; *P<0.05 versus the blank, mimics NC, or inhibitors NC groups; #*P<*0.05 versus the miR-148a inhibitors + siRNA-NC group; &*P<*0.05 versus the miR-148a inhibitors + RRS1 siRNA group; there are six parallel wells in each experiment; the data represent the mean ± S.D. of the three independent experiments.

### Up-regulation of miR-148a inhibits cell cycle progression and induces cell apoptosis in Caski and HeLa cells

Cell cycle distribution and cell apoptosis were detected by flow cytometry. The results of cell cycle detection of Caski (Figure 7A) and HeLa (Figure 7C) cells by PI single staining showed that in Caski (Figure 7B) and HeLa (Figure 7D) cells, in contrast with the blank, mimics NC and inhibitors NC groups, more cells arrested at G0/G1 phase and fewer cells in S phase in the miR-148a mimics and RRS1 siRNA groups while fewer cells arrested at G0/G1 phase and more cells in S phase in the miR-148a inhibitors and miR-148a inhibitors + siRNA-NC groups (all *P<*0.05). No significant difference was found in cell cycle distribution amongst the blank, mimics NC and inhibitors NC groups (*P*>0.05). In comparison with the miR-148a inhibitors + siRNA-NC group, more cells arrested at G0/G1 phase and fewer cells in S phase in the miR-148a inhibitors + RRS1 siRNA group (*P<*0.05). There was no significant difference in cell distribution of G2/M in each group (*P*>0.05). Compared with the miR-148a inhibitors + RRS1 siRNA group, more cells arrested at G0/G1 phase and fewer cells in S phase in the RRS1 siRNA group (*P<*0.05). It is further suggested that in Caski and HeLa cells, up-regulation of miR-148a inhibits cell cycle progression.

**Figure 7:** Up-regulation of miR-148a inhibits cell cycle progression in Caski and HeLa cells (**A,B**) Cell cycle distribution of Caski cells in each group; (**C,D**) cell cycle distribution of HeLa cells in each group; *P<0.05 versus the blank, mimics NC, or inhibitors NC groups; #*P<*0.05 versus the miR-148a inhibitors + siRNA-NC group; &*P<*0.05 versus the miR-148a inhibitors + RRS1 siRNA group; there are six parallel wells in each experiment; the data represent the mean ± S.D. of the three independent experiments.

Annexin-V-FITC and PI double staining was applied to detect the apoptosis of Caski (Figure 8A) and HeLa (Figure 8C) cells. As shown in Figure 8, in Caski (Figure 8B) and HeLa (Figure 8D) cells, in contrast with the blank, mimics NC, and inhibitors NC groups, cell apoptosis rate was increased in the miR-148a mimics and RRS1 siRNA groups while decreased in the miR-148a inhibitors and miR-148a inhibitors + siRNA-NC groups (all *P<*0.05). No significant difference was found in cell apoptosis rate amongst the blank, mimics NC and inhibitors NC groups (*P*>0.05). In comparison with the miR-148a inhibitors + siRNA-NC group, cell apoptosis rate was increased in the miR-148a inhibitors + RRS1 siRNA group (*P<*0.05). Compared with the miR-148a inhibitors + RRS1 siRNA group, the RRS1 siRNA group showed increased cell apoptosis rate (*P<*0.05). The results suggested that in Caski and HeLa cells, up-regulation of miR-148a promotes cell apoptosis.

**Figure 8:** Up-regulation of miR-148a induces apoptosis of Caski and HeLa cells (**A,B**) Cell apoptosis of Caski cells in each group; (**C,D**) cell apoptosis of HeLa cells in each group; *P<0.05 versus the blank, mimics NC, or inhibitors NC groups; #*P<*0.05 versus the miR-148a inhibitors + siRNA-NC group; &*P<*0.05 versus the miR-148a inhibitors + RRS1 siRNA group; there are six parallel wells in each experiment; the data represent the mean ± S.D. of the three independent experiments.

### Up-regulation of miR-148a suppresses migration of Caski and HeLa cells

Cell scratch test was performed to assess the migration of Caski (Figure 9A) and HeLa (Figure 9C) cells. The results showed that in Caski (Figure 9B) and HeLa (Figure 9D) cells, in contrast with the blank, mimics NC, and inhibitors NC groups, the healing rate was decreased in the miR-148a mimics and RRS1 siRNA groups while increased in the miR-148a inhibitors and miR-148a inhibitors + siRNA-NC groups (all *P<*0.05). No significant difference was found in the healing rate amongst the blank, mimics NC and inhibitors NC groups (*P*>0.05). In comparison with the miR-148a inhibitors + siRNA-NC group, healing rate was decreased in the miR-148a inhibitors + RRS1 siRNA group (*P*<0.05). Compared with the miR-148a inhibitors + RRS1 siRNA group, the RRS1 siRNA group showed decreased healing rate (*P<*0.05).The results suggested that in Caski and HeLa cells, up-regulation of miR-148a inhibits cell migration.

**Figure 9:** Up-regulation of miR-148a suppresses migration of Caski and HeLa cells Note: (**A-B**) Scratch gap fusion of Caski cells in each group; (**C,D**) scratch gap fusion of HeLa cells in each group; *P<0.05 versus the blank, mimics NC, or inhibitors NC groups; #*P<*0.05 versus the miR-148a inhibitors + siRNA-NC group; &*P<*0.05 versus the miR-148a inhibitors + RRS1 siRNA group; there are six parallel wells in each experiment; the data represent the mean ± S.D. of the three independent experiments.

### Up-regulation of miR-148a suppresses invasion of Caski and HeLa cells

Transwell assay was conducted to detect the invasion of Caski (Figure 10A) and HeLa (Figure 10C) cells. The results showed that in Caski (Figure 10B) and HeLa (Figure 10D) cells, compared with the blank, mimics NC, and inhibitors NC groups, the number of invasive cells was decreased in the miR-148a mimics and RRS1 siRNA groups while which was increased in the miR-148a inhibitors and miR-148a inhibitors + siRNA-NC groups (all *P*<0.05). No significant difference was found in the number of invasive cells amongst the blank, mimics NC, and inhibitors NC groups (*P*>0.05). In contrast with the miR-148a inhibitors + siRNA-NC group, the number of invasive cells was decreased in the miR-148a inhibitors + RRS1 siRNA group (*P<*0.05). Compared with the miR-148a inhibitors + RRS1 siRNA group, the RRS1 siRNA group showed decreased number of invasive cells (*P*<0.05). The results demonstrated that in Caski and HeLa cells, up-regulation of miR-148a inhibits cell invasion.

**Figure 10:** Up-regulation of miR-148a suppresses invasion of Caski and HeLa cells (**A,B**) Invasion ability of Caski cells in each group; (**C,D**) invasion ability of HeLa cells in each group; *P<0.05 versus the blank, mimics NC, or inhibitors NC groups; #*P<*0.05 versus the miR-148a inhibitors + siRNA-NC group; &*P<*0.05 versus the miR-148a inhibitors + RRS1 siRNA group; there are six parallel wells in each experiment; the data representsthe mean ± S.D. of the three independent experiments.

## Discussion

Accumulating evidence has suggested that miRNAs play vital roles in many kinds of human malignant cancers including cervical cancer [26]. Several miRNAs, such as miR-182, miR-1246, and miR-29a, have been demonstrated to be involved in cervical cancer [27–29]. In consideration of the relationship between miR-148a and RRS1, we suspected that miR-148a might play a pivotal role in cervical cancer. In the present study, we found that miR-148a was lowly expressed in cervical cancer, and up-regulated miR-148a significantly inhibited the expression of RRS1. Besides, up-regulation of miR-148a inhibited the proliferation, migration, and invasion as well as induced apoptosis of cervical cancer cells. Thus, our study might provide new insights into the pathogenesis and strategies for cervical cancer treatment.

One of the most significant findings in our study was that down-regulated miR-148a and up-regulated RRS1 were found in cervical cancer tissues and cells. In accordance with the results in our study, a previous study has found that compared with non-tumorous controls, highly expressed miR-152 and miR-148a are found in gastrointestinal cancer tissues and cells [30]. It has also been suggested that down-regulated miR-148a expression is detected in several types of cancer, including prostate cancer [31], pancreatic ductal adenocarcinoma [32], and hepatoblastoma [33]. Meanwhile, numerous studies have revealed that down-regulation of miR-148a is found in various types of human cancer, such as gastric cancer, breast cancer, hepatocellular carcinoma, as well as pancreatic ductal adenocarcinoma, which is regarded as a tumor-suppressive miRNA [34–37]. As for the RRS1, the RRS1 mRNA expression in hepatocellular carcinoma (HCC) tissues was significantly higher than that in adjacent tissues, and the up-regulation of RRS1 may play an essential role in the pathogenesis of HCC [38].

Additionally, our study also found that RRS1 was a target gene of miR-148a and miR-148a inhibited RRS1 expression in cervical cancer cells. So far, previous studies have demonstrated that the direct target genes of miR-148a include MSK1, TGIF2, DNMT3, as well as PXR [31, 38–40]. However, the functional roles together with target genes of miR-148a in cervical cancer have not yet been uncovered. The present study showed that RRS1 is a direct target gene of miR-148a in cervical cancer Caski and HeLa cells. Meanwhile, the tumor suppressive effects of miR-148a could be controlled by the down-regulation of RRS1 expression.

Furthermore, we also found that up-regulation of miR-148a inhibited proliferation, migration, and invasion while promoting apoptosis in Caski and HeLa cells. MiR-148a is a member of the miR-148 family, and it had close correlation with diverse biological functions, such as proliferation, migration, invasion, as well as cell cycle progression [41–43]. Besides, miR-148a functions as a tumor suppressor in multiple types of tumors in order to block the growth and metastasis of cells [44–46]. Zhou et al. have demonstrated that miR-148a was poorly expressed in ovarian cancer cells and whose overexpression inhibited cell proliferation [47]. Meanwhile, Zheng et al. have proposed that miR-148a is able to inhibit cell invasion and migration in gastric cancer cells by down-regulating ROCK1 [48]. Additionally, it is reported that miR-148a enables to induce apoptosis of colorectal cancer cells through the inhibition of Bcl-2 expression [49]. Besides, overexpression of miR-148a suppressed proliferation, migration, and invasion in gastric cancer cell lines by decreasing expression of TGFβ2 and SMAD2 [50]. Moreover, up-regulated miR-148b expression is capable of protecting against cervical cancer by inducing apoptosis via caspase-3-dependent manner, and up-regulation of miR-148b might provide a therapeutic intervention for cervical cancer [51]. All these aforementioned findings imply a tumor suppressor role for miR-148a in the modulation of tumor progression.

In summary, our study suggests that miR-148a down-regulates RRS1 expression, thereby inhibiting the proliferation, migration, and invasion while promoting apoptosis of cervical cancer cells, suggesting that miR-148a may be a novel biomarker for early detection or therapeutic targets of cervical cancer. In the future, we would prolong the follow-up time, and study the other target genes of miR-148a, so as to establish the foundation for further study on the function of miR-148a.

## Abbreviations

FBS: fetal bovine serum
GAPDH: glyceraldehyde-3-phosphate dehydrogenase
HCC: hepatocellular carcinoma
NC: negative control
OD: optical density
PI: propidium iodide
RRS1: ribosome synthesis 1
RT-qPCR: reverse transcription quantitative PCR
